The article "Immunoregulation and antidepressant effect of ketamine" was published in 2021. Journal: Transl Neurosci.

# Immunoregulation and antidepressant effect of ketamine

**DOI:** 10.1515/tnsci-2020-0167

**Published:** 2021-05-26

**Authors:** Nan Zhang, Lihua Yao, Peilin Wang, Zhongchun Liu

**Affiliations:** Department of Psychiatry, Renmin Hospital of Wuhan University, Jiefang Rd. 238, 430060, Wuhan, China

**Keywords:** ketamine, depression, antidepressant therapy, cytokine, neuroimmunity, NMDAR

## Abstract

Major depressive disorder (MDD) is a common mental health disorder that brings severe disease burden worldwide. Traditional antidepressants are mainly targeted at monoamine neurotransmitters, with low remission rates and high recurrence rates. Ketamine is a noncompetitive glutamate *N*-methyl-d-aspartate receptor (NMDAR) antagonist, and its rapid and powerful antidepressant effects have come to light. Its antidepressant mechanism is still unclarified. Research found that ketamine had not only antagonistic effect on NMDAR but also strong immunomodulatory effect, both of which were closely related to the pathophysiology of MDD. Although there are many related studies, they are relatively heterogeneous. Therefore, this review mainly describes the immune mechanisms involved in MDD and how ketamine plays an antidepressant role by regulating peripheral and central immune system, including peripheral inflammatory cytokines, central microglia, and astrocytes. This review summarizes the related research, finds out the deficiencies of current research, and provides ideas for future research and the development of novel antidepressants.

## 1 Introduction

Major depressive disorder (MDD) is an affective disorder characterized by significant and persistent low mood, anhedonia, and activity decline. The high morbidity, recurrence rate, and disability rate of MDD have led to serious disease burden throughout the world [1]. However, the pathogenesis of MDD has not been fully elucidated. Currently, pharmacological therapy is mainly targeted at monoamine neurotransmitters, yet which have low remission rates (no symptomatic remission rates are up to 40% even after twice treatments), have slow effects (6–8 weeks or longer to obtain response or remission), and high recurrence rates [2–5]. Therefore, there is an urgent need to find drugs that work faster and more effectively through other mechanisms [6,7]. Although the treatment of MDD with monoaminergic antidepressants is still unsatisfactory, the inhibitors of both norepinephrine and serotonin transporters (SNRIs) have tested their efficacy in acute MDD. In particular, duloxetine has good evidence of efficacy in acute, adult MDD, especially at doses of 80–120 mg/day [8]. In addition, agomelatine, a melatonin analog, is of particular interest due to another alternative mechanism of action. The clinical efficacy, safety, and tolerability of this compound have been widely confirmed. Agomelatine enhances neuroplasticity mechanisms and adult neurogenesis in brain areas such as hippocampus and prefrontal cortex [9]. Animal research also showed that treatment with agomelatine reversed the signs of anxiety and depression, and decreased the cytokines (tumor necrosis factor-α [TNF-α], interleukin 6 [IL-6], and IL-1β), thiobarbituric acid reactive substances, as well as caspase-3 activity [10]. The anti-inflammatory activities of both duloxetine and agomelatine have been found to be correlated with the tryptophan metabolism pathway [11]. These studies suggest that the antidepressant effect of antidepressants may be related to their anti-inflammatory mechanism. In recent years, it has been found that subanesthesia dose of ketamine produced a notable, rapid, and lasting antidepressant effect when used for patients with MDD including treatment-resistant depression (TRD) [12,13,14]. Ketamine is a noncompetitive glutamate *N*-methyl-d-aspartate receptor (NMDAR) antagonist. Studies have found that its antidepressant mechanism involved not only glutamate inhibitory pathway, α-amino-3-hydroxy-5-methyl-4-isoxazolyl propionic acid (AMPA) receptor signal pathway, and neural plasticity but also immune regulation, including peripheral and central immune regulations [15].

The article "Immunoregulation and antidepressant effect of ketamine" was published in 2021. Journal: Transl Neurosci.

This study mainly summarizes the relationship between MDD and immune dysregulation, and the immunomodulatory mechanism of the antidepressant effects of ketamine, in order to provide ideas for the development of novel antidepressants with more effective and less side effects in the future.

We conducted a narrative review of available literature up to July 2020 using PubMed, Elsevier, and Web of Science. The search terms were as follows: “major depressive disorder,” “depression,” “mood disorder,” “cytokine,” “inflammation,” “chemokine,” “neuroimmunity,” “immune,” “ketamine,” “esketamine,” “NMDAR,” “Glutamate receptor,” and “Glutamate.” We selected studies based on their overall methodological quality, whether they fit the topic of the article, and how comprehensive and innovative they were. We included not only original research in human and animal models but also reviews and book chapters.

## 2 Immune dysregulation and depression

Plenty of studies have shown that immune dysfunction was involved in the pathophysiology of MDD. Many case–control studies had identified that many pro-inflammatory cytokines, such as IL-6, and C-reactive protein (CRP), increased in MDD compared to healthy controls [16,17]. A cohort study followed up for 6 years discovered that higher baseline levels of plasma IL-6 predicted chronic recurrent course in women with MDD, and cytokines were expected to be biomarkers for predicting recurrence of depression [18]. Several meta-analyses have indicated that depressive patients had higher pro-inflammatory cytokines, such as IL-6 and TNF-α, suggesting that inflammation may be involved in the pathogenesis of MDD [19,20,21]. A large number of studies have demonstrated that pro-inflammatory cytokines usually increased in MDD, among them IL-6, TNF-α, and interferon γ (INF-γ) were found relatively consistent [22]. However, some research on anti-inflammatory and other cytokines in MDD are inconsistent. Clinical studies found that IL-5, IL-15, IL-10, IL-2, and IL-13 increased and IL-1 receptor antagonist, IL-4 decreased, while a meta-analysis showed that IL-2, IL-4, and IL-10 unchanged. The heterogeneity may be related to confounding factors (such as subjects’ average age and body mass index), and some studies have shown that depression was not associated with peripheral inflammation after controlling confounding factors [23,24]. Recently, the changes in immune cells in MDD have also been concerned. For example, a case–control study found that depression cases, compared with controls, had significantly increased immune cell counts, especially neutrophils, CD4^+^ T cells, and monocytes [16]. The research also implied that peripheral immune cell counts could be used to distinguish inflamed and uninflamed subgroups of depression and to indicate that there might be mechanistically distinct subgroups of inflamed depression [16]. This study lists several previous clinical studies and meta-analysis on the relationship between immune disorders and depression in Table 1 to provide relevant information for researchers.

The article "Immunoregulation and antidepressant effect of ketamine" was published in 2021. Journal: Transl Neurosci.

**Table 1:** Immune dysregulation and depression

Study design	Subjects	Sample size	Biomarkers	Case vs control	Correlation between inflammatory factors and depression	Reference
Meta-analysis	MDD vs HCs	N/A	Peripheral blood IL-6, TNF-α, IL-10, sIL-2R, CCL-2, IL-13, IL-18, IL-12, IL-1Ra, sTNFr2	MDD (vs HCs) ↑	Not available	[20]
			INF-γ	MDD (vs HCs) ↓		
Meta-analysis	MDD vs HCs	N/A	Peripheral blood sIL-2R, TNF-α, IL-6	MDD (vs HCs) ↑	Not available	[21]
			IL-1β, IFN-γ, IL-2, IL-4, IL-8, IL-10	MDD (vs HCs) NS		
Cross-sectional and bidirectional longitudinal associations	Current depressive disorder in the past 6 months (CDS), no current disorder, with and without a prior history of MDD (NCDS)	The baseline (*n* = 2,416) and 2- and 6-year follow-up assessments (*n* = 1,925 and *n* = 1,924, respectively)	Fasting morning blood plasma IL-6	Baseline CDS (vs no current disorder) ↑	Cross-sectional positive associations between depression and IL-6 over three waves; in longitudinal analyses, higher baseline IL-6 levels predicted higher depression at follow-up in women but not in men, and both depressive disorder and high severity predicted higher IL-6 levels at the subsequent follow-up	[18]
			CRP	Baseline CDS (vs NCDS) NS	C-reactive protein was not associated with current depression in cross-sectional and longitudinal analyses	
Meta-analysis	MDD vs controls (psychiatrically healthy subjects)	N/A	TNF-α, IL-6	MDD (vs controls) ↑	Not available	[23]
			IL-1β, IL-4, IL-2, IL-8, IL-10, INF-γ	MDD (vs controls) NS		
Meta-analysis	MDD vs controls (included studies with participants suffering from physical comorbidity)	N/A	Blood CXCL4, CXCL7	MDD vs controls (included participants suffering from physical comorbidity) ↑		[31]
			Blood CCL4	MDD vs controls (included participants suffering from physical comorbidity) ↓		
			Blood CCL2, CCL3, CCL11, CXCL8, CCL5, CCL7, CXCL9, CXCL10, and cerebrospinal fluids CXCL8 and CXCL10	MDD vs controls (included participants suffering from physical comorbidity) NS		
			Blood levels of CCL2, CCL3, CCL11, CXCL4, CXCL7, and CXCL8	MDD vs controls (only physically healthy participant) ↑		
			CCL4	MDD vs controls (only physically healthy participant) ↓		
			Blood CCL5, CCL7, CXCL9, CXCL10, and cerebrospinal fluids CXCL8 and CXCL10	MDD vs controls (only physically healthy participant)		
Cross-sectional and longitudinal associations	Treatment-naive MDD vs HCs	Baseline cytokines MDD (*n* = 171), HC (*n* = 64), Baseline Inflammasome Protein MDD (*n* = 24), HC (*n* = 24), activated PBMCs HC (*n* = 27) MDD (*n* = 40)	IL-12, TNF, IL-6, IFN-γ, IL-9, IL-17A, IL-5, IL-15, IL-10, IL-2, IL-13, MIP1α/CCL3, RANTES, Caspase-1, IL-18, ASC1	MDD (vs HCs) ↑	Not available	[24]
			CCL5, G-CSF, PDGF, FGF, IL-7, IL-1Ra, IL-4, MIP1β/CCL4, IL-8, MCP-1/CCL2, IP-10/CXCL10,CD4+ CD45RO+ CD69−, CD19+CD69+, CD11b+CD86+	MDD (vs HCs) ↓		
			IL-1β, Eotaxin/CCL11, GM-CSF, VEGF, CD4+CD25+CD69+, CD4+CD69+CD45RO-, CD8+CD69+	MDD (vs HCs) NS		
Case–control	Current depression, with or without another comorbid psychiatric disease (i.e. BD, PTSD) vs HCs	Depression on (*n* = 43), HC (*n* = 51)	Blood IL-6	PG (vs HCs) ↑	Correlations between TNF-α and depressive symptoms were found	[17]
			IL-1β, CRP, TNF-α, and IFN-γ	PG (vs HCs) NS		
Case–control	Depression cases (current or past depressive symptoms) and age- and sex-matched controls	Depression on (*n* = 206), HC (*n* = 77)	CRP, IL-6, absolute counts of neutrophils, intermediate monocytes, and CD4^+^ (helper) T cells	PG (vs HCs) ↑	Correlations between neutrophils, CD4^+^ (helper) T cells, CRP, and depressive symptoms were found	[16]
			Eosinophils, basophils, lymphocytes, monocytes, red blood cells, and platelets, CD8^+^ T cells, B cells, classical monocytes, non-classical monocytes, CD16hi NK cells, CD56hi, NK cells, and NK T [NKT] cells	PG (vs HCs) NS		

MDD, major depressive disorders; HCs, healthy controls; N/A, not applicable; IL, interleukin; TNF, tumor necrosis factor; sIL-2R, soluble interleukin-2 receptor; CCL, C–C chemokine ligand 2; IL-1Ra, IL-1 receptor antagonist; sTNFr2, soluble TNF receptor 2; INF, interferon; CRP, C-reactive protein; CXCL, C-X-C chemokine ligand; RANTES, regulated upon activation normal T-cell expressed and secreted; G-CSF, granulocyte colony-stimulating factor; PDGF, platelet-derived growth factor; FGF, fibroblast growth factor; ASC, apoptosis-associated speck-like protein containing a caspase recruitment domain; MIP, macrophage inflammatory protein; MCP-1, monocyte chemoattractant protein-1; PG, patient group; NK, natural killer cell.

The article "Immunoregulation and antidepressant effect of ketamine" was published in 2021. Journal: Transl Neurosci.

The incidence of depression in autoimmune and infectious diseases, such as rheumatoid arthritis, septicemia, and viral hepatitis, was significantly higher than that in healthy controls [25]. To further probe the relationship between cytokines and depression, some researchers have examined patients undergoing treatment with cytokines treatment for multiple sclerosis (MS) and cancers. MS is an autoimmune disease characterized by inflammatory demyelination of the central nervous system (CNS). INF-β is a safe and efficient treatment for MS [26]. Although MS has been found usually accompanied by mental disorders, including depression, Fragoso et al. reported on 11 cases of severe depression with suicide attempts or ideation among patients with MS who were using IFN-β and without previous history of any psychiatric disease. IFN-β withdrawal led to complete remission of symptoms [27]. Other innate immune cytokines, such as IFN-α, in the treatment for cancers, also cause significant depressive symptoms, depending on the dose [28–30]. Therefore, the above data from cytokine treatment for MS and cancers provide a further connection of depression in the immune system.

In addition, chemokines seem to be involved in the occurrence of depression. A meta-analysis assessed chemokine levels in patients with MDD without medical disease and found that peripheral blood CCL2, CCL3, CCL11, CXCL7, and CXCL8 levels were higher and CCL4 levels were lower than control, while no significant differences were found in other chemokines (CCL5, CCL7, CXCL9, CXCL10, and cerebrospinal fluid CXCL8 and CXCL10) [31]. Increasingly, evidence have shown that MDD is closely related not only to cytokines but also to immune cells and chemokines, which further explained that immune dysregulation was deeply involved in the pathophysiology of MDD. Therefore, further study on the immune mechanism of depression may help to find the target of antidepressants in the immune system.

The article "Immunoregulation and antidepressant effect of ketamine" was published in 2021. Journal: Transl Neurosci.

## 3 Immunomodulatory effects of classical antidepressants and ketamine

In this section, we introduce the similarities and differences of immune regulation between classical antidepressants and ketamine.

*In vitro* experiments found that selective serotonin reuptake inhibitors (SSRIs) and tricyclic antidepressants had anti-inflammatory effects. Studies have found that clomipramine, sertraline, and trazodone could reduce INF-γ and increase IL-10 levels *in vitro* [32]. Glial cell culture found that fluoxetine and imipramine treatment can inhibit microglia and reduce culture medium TNF-α and IL-1β levels induced by lipopolysaccharide (LPS) [33]. However, *in vitro* studies cannot confirm that their anti-inflammatory effects are related to antidepressant effects.

Animal research further found that amitriptyline decreased NO production to exert the anti-inflammatory effects [34]. Imipramine treatment reverses depressive- and anxiety-like behaviors, normalizes adrenocorticotropic hormone, and reduces interleukin-1β in the brain of rats subjected to experimental periapical lesion [35]. Previous studies have found that ketamine has a strong anti-inflammatory effect, and cytokines are supposed to be used as biomarkers to predict the antidepressant effect of ketamine [36]. A single dose of ketamine reduced elevatory serum levels IL-1β and IL-6 to normal in depression-like rats caused by neuralgia. We summarize the preclinical research cited in this study in Table 2.

**Table 2:** Preclinical experiments on antidepressants and inflammation

Study design	Types of cells or animals	Sample size	Biomarkers assessed	Conditions	Changes	Drug	Type of treatment	Duration	Effects	Outcome of depression	Reference
Cell culture	Primary rat mixed glial cell	N/A	TNF-α, IL-1β, IL-10, TNF-α mRNA, IL-1β mRNA, NF-κB p65 subunit	LPS-stimulated	↑	Imipramine, fluoxetine	N/A		↓	N/A	[33]
			IL-10 mRNA		↑	Fluoxetine			NS		
						Imipramine			↓		
Animal research	Male Wistar rats	10× group	TNF-α, IL-1β in serum	Carrageenan-induced paw edema (CIPE) and acute peritonitis	Not available	Amitriptyline, L-NAME (a NO synthase inhibitor), or both of amitriptyline, L-NAME	Preventive	3 h	↓	Not available	[34]
			Nitrates, total of leukocytes in serum			Both of amitriptyline, L-NAME			↓		
						Amitriptyline, L-NAME			NS		
Animal research	Male Wistar rats	10 × 2 group	IL-1β, IL-6	Acute stress by a forced swimming test (FST) for 15 min	Not available	A single dose of Ketamine 10 mg/kg	Therapeutic	30 min	↓	Immobility time during FST ↓	[85]
	Male Sprague–Dawley rats		IL-1β, IL-6	Spared nerved ligation (SNI)	↑	A single dose of ketamine (20 mg/kg)	Therapeutic	24 h	↓	Responders (vs nonresponders)↓ both at baseline and after treatment	[36]
			TNF-α		↑				NS	Responders (vs nonresponders) NS both at baseline and after treatment	

TNF, tumor necrosis factor; IL, interleukin; mRNA, messenger RNA; NF-κB, nuclear factor kappa-B; LPS, lipopolysaccharide; FST, forced swimming test; N/A, not applicable; NS, not significant.

The article "Immunoregulation and antidepressant effect of ketamine" was published in 2021. Journal: Transl Neurosci.

Clinical evidence also shows that some antidepressants have anti-inflammatory effects. Meta-analysis evaluated the effects of antidepressants on cytokine levels and found that levels of IL-6 decreased with treatment regardless of outcome, whereas persistently elevated TNF-α was associated with prospectively determined treatment resistance [37]. Other studies have shown that immune markers may be used as predictors of treatment outcomes [38]. It is generally believed that higher cytokine levels are associated with adverse therapeutic responses to monoamine antidepressants. Eller et al. found that when treated with escitalopram, the higher the baseline TNF-α level was, the worse the treatment response would be [38]. O’Brien found that plasma IL-6 and TNF-α in the SSRI resistance group were higher than those in the treatment response group [39], and the levels of TNF-α, sTNF-αR2, and IL-6 in patients with two or more treatment failures were higher than those in patients with fewer failures [40]. A meta-analysis which evaluated plasma cytokine levels and antidepressant response found that compared with nonresponders, responders had lower baseline IL-8 levels, and their TNF-α levels were significantly reduced by antidepressant therapy [41]. A study followed up for 12 weeks found that the mean value of anti-inflammatory cytokines in both treatment responders and nonresponders increased, while only pro-inflammatory cytokines were stable in the responding group and continued to increase in the nonresponding group. It is speculated that the antidepressant treatment response may be related to whether anti-inflammatory factors can suppress the increase in pro-inflammatory factors IL-1β, IL-6, and TNF-α [24].

In addition, adjuvant anti-inflammatory treatments can improve depression. For example, NSAIDs, cytokine inhibitors, minocycline, and P2X7R antagonists can play a synergistic role in antidepressant treatment [42,43]. Although more experiments are still needed to evaluate safety and efficacy and the effect of single-agent treatment, they do show the potential of anti-inflammatory drugs to improve depression.

The article "Immunoregulation and antidepressant effect of ketamine" was published in 2021. Journal: Transl Neurosci.

Compared with classical antidepressants, ketamine has different results. Park et al. surveyed plasma levels of the eight cytokines at baseline and at 230 min, 1 day, and 3 days postketamine in MDD, and they found that ketamine treatment significantly increased IL-6 levels and reduced sTNFR1 levels at 230 min, but changes in cytokines were not associated with improvement in depression [44]. Chen et al. investigated the relevance between the antidepressant effects of a single ketamine and its inflammation inhibitory effect in patients with TRD, and they examined pro-inflammatory factors, including CRP, IL-6, and TNF-α at baseline and at 40 min, 240 min, day 3, and day 7 postinfusion, then analyzed the relationship between them and depressive symptoms across time, and finally found that compared with baseline, TNF-α decreased at 40 and 240 min postinfusion, and the decrease at 40 min was positively correlated with the decrease of depression score on days 4 and 5, while no positive findings were found at other time points [45]. These results may imply that the rapid inhibition of pro-inflammatory cytokines may contribute to the rapid antidepressant effect of ketamine. Yang et al. found among MDD patients who received ketamine that those responded had higher baseline IL-1β and IL-6 levels than those who did not respond, and the levels of IL-6 decreased significantly after treatment [46]. This suggests that baseline levels of pro-inflammatory factors predict different responses to ketamine and classic antidepressants. This may be due to their different anti-inflammatory ability, which requires more experiments under the same conditions (such as age and degree of depressive symptoms).

Park et al. found that IL-6 in active depression or bipolar depression transiently increased within 4 h after ketamine treatment, but it was not related to treatment response [44]. Another study found that ketamine briefly reduced peripheral IL-6 levels, which was also unrelated to antidepressant response [47]. This may be due to the fact that there is an initial modulation of cytokines following ketamine infusion which may indeed be attributed to some of the earlier phases of ketamine’s activity, perhaps the surge in glutamate, all agree that this has no bearing on treatment response. It may be meaningful to further study these patients, even despite a positive treatment outcome, who may still have high levels of circulating peripheral cytokines. Do these patients benefit from adjunct therapy, are they still more severely ill than other patients despite the response? Do treatment response and cytokine level correlate for repeated treatment? There are numerous questions that are not addressed here but are important in terms of provided meaningful clinical information. We summarize the treatment-related clinical studies cited in this study in Table 3.

The article "Immunoregulation and antidepressant effect of ketamine" was published in 2021. Journal: Transl Neurosci.

**Table 3:** Antidepressant therapy and immune regulation

Study design	Subjects	Sample size	Antidepressant (s)	Duration	Cytokine assessed	Baseline		Follow-up vs baseline		Outcome of follow-up	Reference
A meta-analysis	Depressive patients (with unipolar and BPD) and HCs	N/A	N/A	N/A	TNF-α	Case (vs HC)↑	Responders (vs nonresponders) NS	Responders ↓	Nonresponders (NS)	Didn’t report	[37]
					IL-6 (follow-up vs baseline) ↓, no matter, responders or non-responders, CRP	Case (vs HC)↑	Responders (vs nonresponders) NS	Responders (NS)	Nonresponders (NS)	Didn’t report	
Cohort study	MDD (Moderate or severe) vs HCs	MDD (*n* = 100), HC (*n* = 45)	Escitalopram 10–20 mg/day	4, 12 Weeks	TNF-α	Case (vs HC) NS	Responders (vs nonresponders) ↓	Responders (NS)	Nonresponders (NS)	Case (vs HC) NS, responders (vs nonresponders) NS	[38]
					sIL-2R	Case (vs HC) NS	Responders (vs nonresponders) NS	Responders ↓ at 4 weeks	Nonresponders (↓ both at 4 and 12 weeks)	Case (vs HC) NS, responders (vs nonresponders) NS	
					IL-8	Case (vs HC) NS	Responders (vs nonresponders) NS	Responders (NS)	Nonresponders (NS)	Case (vs HC) NS, responders (vs nonresponders) NS	
Cross-sectional	28 MDD (19 fe, 9 m) with HAMD-17 > 20 who had failed a 6-weeks course of an SSRI, 16 subjects (11 fe, 5 m) previously SSRI resistant but now euthymic (HAMD-17 < 8), 24 healthy comparison subjects (14 fe, 10 m), age from 25 to 55 years		Fluoxetine, paroxetine or citalopram at a minimum of 20 mg daily	N/A	IL-6, TNF-α	N/A	N/A	N/A	N/A	Current (vs both previously SSRI resistant and HCs) ↑, **SSRI resistant vs HCs (NS)**	[39]
					IL-8, IL-10, sIL-6R	N/A	N/A	N/A	N/A	Current SSRI resistant vs previously SSRI resistant vs HCs (NS)	
Cross-sectional	Unmedicated, medically stable patients with MDD and varying numbers of adequate antidepressant treatment trials in the current depressive episode, ages of 21 and 65 years, *n* = 98			N/A	IL-6, TNF-α, sTNF-R2	N/A	N/A	N/A	N/A	Patients with 3 or more failed trials in the current episode (vs individuals with 0 or 1 trial) ↑ CRP was also associated with a greater number of treatment failures, but only in models with BMI excluded.	[40]
					CRP	N/A	N/A	N/A	N/A		
A meta-analysis	MDD vs HCs or MDD responders vs MDD nonresponders	N/A	N/A	At least 4 weeks	IL-8	N/A	Responders (vs nonresponders) ↓	Responders (NS)	Nonresponders (NS)	Responders (vs nonresponders) NS	[41]
					TNF-α	N/A	Responders (vs nonresponders) NS	Responders ↓	Nonresponders (NS)	Responders (vs nonresponders) ↓	
					GM-CSF	N/A	Responders (vs nonresponders) NS	Responders ↓	Nonresponders (NS)	Responders (vs nonresponders) NS	
					IL-5	N/A	Responders (vs nonresponders) NS	Responders ↓	Nonresponders ↓	Responders (vs nonresponders) NS	
					IL-1β, IL-2, IL-4, IL-6, IL-10, IL-12, CRP, IFN-γ, GM-CSF, MIP-1α 和Eotaxin-1	N/A	Responders (vs nonresponders) NS	Responders (NS)	Nonresponders (NS)	Responders (vs nonresponders) NS	
Cohort study	171 Baseline treatment-naive MDD vs 64 HCs		Escitalopram (10–20 mg/day), duloxetine (30–60 mg/day), or 16 sessions of CBT of 50 min	12 Weeks	IL-6, IFN-γ, IL-1β, TNF, IL-17A	Discussed in Table 1	Responders (vs nonresponders) not available	Responders (NS)	Nonresponders ↑	Responders (vs nonresponders) not available	[24]
	Follow-up Responder (*n* = 33), nonresponder (*n* = 71)				IL-2, IL-4, IL-5, IL-10, IL-15	Discussed in Table 1	Responders (vs nonresponders) not available	Responders ↑	Nonresponders ↑	Responders (vs nonresponders) not available	
Meta-analysis	Patients with ketamine before or during operation	N/A	Ketamine	N/A	IL-6	N/A	N/A	↓		N/A	[86]
A randomized, double blind control study	71 TRD patients		0.5 mg/kg ketamine, 0.2 mg/kg ketamine, and normal saline infusion	Single	CRP, IL-6	0.5 mg/kg ketamine vs 0.2 mg/kg ketamine vs normal saline infusion (NS)	N/A	NS at 40 min, 240 min, day 3, and day 7 postinfusion		NS correlation between them and depression	[45]
					TNF-α	0.5 mg/kg ketamine vs 0.4 mg/kg ketamine vs normal saline infusion (NS)	N/A	↓ at 40 min and 240 min after 0.5 mg/kg ketamine infusion		Decrease at 40 min was positively correlated with the decrease of depression score on day 4 and day 5	
A double-blind, placebo-controlled study	MDD or BD (*n* = 80)		0.5 mg/kg ketamine	Single	IL-6	MDD (vs BD) ↓	NS correction between IL-6 with BS depression	↑		NS correlation between them and depression	[44]
					TNF-α	MDD (vs BD) ↓	NS correction between TNF-α with BS depression	NS		NS correlation between them and depression	
					sTNFR1	MDD (vs BD) ↑	sTNFR1 was positive correction with BS depression	↓		NS correlation between them and depression	
					IFN-g, IL-2, IL-5,IL-8, and IL-10	MDD (vs BD) NS	NS correction between TNF-α with BS depression	NS		NS correction between TNF-α with BS depression	
Cohort study	MDD patients were antidepressant-free for at least 2 weeks, healthy volunteers	MDD (*n* = 16), HCs (*n* = 24)	Ketamine	Single	IL-1β	case (vs HC) ↑	Responders (vs nonresponders) ↑	Responders ↓ at 230 min and 1 day	Nonresponders (NS)	Didn’t report	[46]
					IL-6	Responders (vs HC) ↑, nonresponders (vs HC)NS	Responders (vs nonresponders) ↑	Responders ↓ at 230 min and 3 days	Nonresponders (NS)		
					TNF-α	Case (vs HC) ↑	Responders (vs nonresponders) ↑	Responders (NS)	Nonresponders (NS)		

N/A, not applicable; MDD, major depressive disorders; HCs, healthy controls; IL, interleukin; TNF, tumor necrosis factor; CRP, C-reactive protein; NS, not significant; sIL-2R, soluble interleukin-2 receptor; SSRI, selective serotonin reuptake inhibitor; sIL-6R, soluble interleukin-6 receptor; fe, female; m, male; sTNFr2, soluble TNF receptor 2; INF, interferon; GM-CSF, granulocyte-macrophage colony-stimulating factor; MIP, macrophage inflammatory protein.

The article "Immunoregulation and antidepressant effect of ketamine" was published in 2021. Journal: Transl Neurosci.

## 4 Pathophysiological mechanism of cytokines involved in depression

Rodent animal studies have found that injection of cytokines can induce depressive symptoms such as behavioural despair, and psychomotor retardation [48]. LPS is the main component of the cell wall of Gram-negative bacteria [49]. LPS can bind with serum lipopolysaccharide-binding protein (LBP) to form LPS/LBP compound, which acts on immune cell membrane receptor CD14 or soluble CD14 to produce a series of biological effects, including inflammatory response [50–52]. LPS can increase the level of IL-1β and IL-6 in prefrontal cortex and lead to depression-like behavior in rats [53].

Interferon superfamily plays a role in host-defense mechanisms. Interferons are usually prescribed to treat various autoimmune (e.g., MS), viral (e.g., chronic hepatitis B and C), and malignant (e.g., malignant melanoma and hairy cell leukemia) disorders [54]. IFN therapy (α, β) induces hypothalamus–pituitary–adrenal (HPA) axis hyperactivity, which is conventionally associated with risk of depression [55]. IFN-α is suggested to modulate mood by the activation of the pro-inflammatory cytokines that comprise IFN-induced 15 kDa protein, ubiquitin-specific proteinase 18, guanylate-binding protein 3, IL-1, L-6, TNF-α, caspase-4, and caspase-8 or death-activating protein kinases. In addition, IFN-α and IFB-β can activate μ opioid receptor, which increases prostaglandin E2 levels in brain, in turn increases the indoleamine-2,3-dioxygenase (IDO) pathway, which leads to neurotoxicity, finally develops depression [48,55].

Bacillus Calmette–Guerin vaccine (BCG), with immunomodulatory function, has been used to prevent tuberculosis [56]. BCG, like INF, has also been suspected to induce depression due to its effects in IDO induction and kynurenine (KYN) pathway metabolism [57]. This effect might be related to the increase in IL-6 and INF-γ [57,58]. The aforementioned studies may indicate that the disorder of IDO system is related to depression caused by exogenous inflammatory factors. Inflammatory factors such as IL-1, INF-γ, and TNF-α can highly induce the activation of IDO, reduce the degradation of tryptophan to 5-HT, and increase its conversion to KYN. Two hypotheses regarding the upregulation of KYN in the pathogenesis of MDD have been proposed. First, the upregulation of KYN will reduce the bioavailability of tryptophan for the synthesis of 5-HT. Second, the metabolism of KYN can eventually produce 3-hydroxykynurenine and quinolinic acid (Quin) increasing the formation of reactive oxygen species involved in neuronal processes and inducing overstimulation of NMDARs, which lead to hippocampal damage and development of MDD, respectively [59]. Quin also inhibits glutamate reuptake in the astrocyte, thereby increasing synaptic glutamate. It is believed that excessive extracellular glutamate is the main source of excitotoxicity, which is also the cause of apoptosis and neurodegenerative diseases [60]. Therefore, inhibition of excessive inflammation and IDO pathway can reduce neurotoxicity by reducing the excessive increase of extrasynaptic glutamate and NMDAR activation, thereby improve depressive symptoms. Cytokines can participate in the pathogenesis of MDD through the metabolism of monoamine neurotransmitters and various amino acids (tyrosine, tryptophan, phenylalanine, and glutamic acid). The effects of various cytokines on emotion may be achieved through their interaction with the CNS: (1) inflammatory cytokines (such as IL-1β) or peripheral blood mononuclear cells (PBMCs) can act on the vagus nerve, which directly projects to multiple brain regions [61]; (2) peripheral cytokines can spread to the ventricles and choroid plexus of the CNS by volume diffusion [62]; (3) CNS also partly participates in the process of peripheral cytokines and inflammatory cells entering the center. Microglia and astrocytes produce CCL-2 chemotactic monocytes into the brain; and (4) interaction between gut microbiota and CNS affects inflammation [63]. Peripheral inflammatory stimulus activate P38 mitogen-activated protein kinase, thereby increasing 5-HT reuptake, leading to depression [64]; pro-inflammatory cytokines can also reduce tetrahydrobiamine (BH4) availability, BH4 is a key coenzyme factor in monoamine synthesis [65]. IFN-α is associated with decreased peripheral conversion of Phen to Tyr, which in turn is associated with reduced DA in the brain as well as fatigue [66]; hr-CRP > 3 mg/L is related to the increase in glutamate in the basal ganglia, which is related to the anhedonia and psychomotor retardation in MDD [67].

The article "Immunoregulation and antidepressant effect of ketamine" was published in 2021. Journal: Transl Neurosci.

In addition, toll-like receptors (TLRs) are also involved in the pathogenesis of depression, especially the activation of TLR4 in the brain. Several studies have found that both acute and chronic stress could activate TLR4-signaling pathways and induced depression-like behavior in rodents [68]. The activation of TLR4 is dependent on myeloid differentiation factor 88 and TIR-domain-containing adapter-inducing interferon-β. The recruitment of these two linker proteins activates the transcription factors, nuclear factor kappa-B, transcriptional activator AP-1, and interferon regulatory factor 3, induces production of the pro-inflammatory factors IL-β, TNF-α, IL-6, and CXCL10, upregulates the expression of COX-2, eventually activates the inflammatory response, and participates in the pathogenesis of MDD [69].

NOD-like receptor protein 3 and purinergic ligand-gated ion channel 7 receptor (P2X7R) play important roles in immunity of CNS. Several studies have shown that P2X7R activation may lead to the activation of microglia. Microglia are the main immune cells of the CNS. Overactivated microglia can release pro-inflammatory and oxidative stress toxicity factors, such as TNF-α, IL-1β, IL-6, and ROS [70]. The P2X7R gene is a susceptible locus for affective disorders, and its knockout has an antidepressant effect in mice. In addition, studies have shown that M1/M2 microglial polarization disorder and T-helper (TH)1/TH2/TH17 imbalance are also involved in the occurrence of depression [71].

The involvement of chemokines in the occurrence of depression may be related to the following mechanisms: CCL2 participates in monocyte migration; CCL2, CCL3, and CXCL10 take part in the changes of neurotransmission and cognitive function [31,72,73]; CXCL8 and CXCL10 are involved in neuroendocrine regulation, which is related to the change in HPA axis function [31,74]. Previous studies have found that when the body is under stress conditions, the HPA axis is activated and the release of glucocorticoids is increased for mobilizing energy storage. However, if the HPA axis is in hyperfunction for a long time, it will lead to hippocampal injury and depression [75–77]. CXCL12-CXCR4 axis may play a role in neurogenesis. Imaging studies found that the volume of frontal lobe, prefrontal cortex, hippocampus, and amygdala in patients with depression decreased and their neurogenesis decreased [78]. CX3CR1 and CX3CL1 are involved in key pathways of communication between microglia and neurons [79].

## 5 Immunoregulatory mechanism of ketamine’s antidepressant function

The classic antidepressant mechanism of ketamine is mainly related to the reward circuit and neural plasticity: (1) regulating glutamate content in the brain by blocking NMDAR; (2) inhibiting cluster firing of lateral habenula nucleus (antireward center) [80]; (3) activating AMPA receptor, blocking elongation factor 2 kinase of eukaryotic cells, increasing release of brain-derived neurotrophic factor (BDNF) and expression of tropomyosin receptor kinase B, inducing mammalian target of rapamycin-signaling pathway and extracellular regulatory protein kinase activation, and improving neuroplasticity [81–84] (Figure 1).

The article "Immunoregulation and antidepressant effect of ketamine" was published in 2021. Journal: Transl Neurosci.

**Figure 1:** Proposed mechanisms of ketamine action as an antidepressant. LPS or psychological stress can induce depression by increasing peripheral and central inflammation. First, they can activate TLRs and NLPR3 through PBMCs, and then they activate innate immune system, such as PBMCs, NK can release pro-inflammatory cytokines (IL-6, TNF-α, IL-1β), which can interact with the central nervous system (CNS) by the four approaches described above (vagus nerve, volume diffusion, CCL-2, and gut microbiota). They can highly induce the activation of IDO, reduce the degradation of tryptophan to 5-HT, and increase its conversion to KYN. First, the upregulation of KYN will reduce the bioavailability of tryptophan for the synthesis of 5-HT; second, the metabolism of KYN can eventually produce Quin, increasing the formation of reactive oxygen species involved in neuronal processes and inducing overstimulation of NMDARs. Ketamine can decrease peripheral inflammation, prevent quin from binding to NMDAR, attenuate morphological microglia reactivity and cytotoxic microglia polarization, reduce the production of quin in microglia, and improve the function of astrocytes.

Studies in humans and animals have found that the rapid antidepressant effect of ketamine involved not only simple anti-inflammatory effects but also more complex immunoregulatory mechanisms [85,86].

For example, ketamine has anti-inflammatory properties in the treatment of MDD, which can polarize macrophages to an M2-like phenotype [87]. Ketamine also decreases gene expressions of macrophage TNF-α, IL-6 [88], and IL-1β [89]. Another study found that ketamine’s potential antisuicidal mechanism was related to the interruption of the KYN pathway, directly or indirectly prevented the increase in pro-inflammatory cytokines, regulated the hyperglutamate state, and increased normal serotonin levels [90].

In summary, in animal experiments, most results show that ketamine can play an antidepressant role by reducing inflammatory factors, but clinical experiments are inconsistent, which may be due to the difficulty of controlling the homogeneity of patients and the small sample size. In addition, most animal models of depression are induced by LPS or stress, both of which can cause inflammation, and there may not be stress factors among clinical patients. Therefore, the antidepressant effect of ketamine due to its anti-inflammatory effect may be stress or LPS dependent. In order to clarify the effect of ketamine and inflammation on TRD, it is necessary to conduct a large sample study in a well-defined population.

The article "Immunoregulation and antidepressant effect of ketamine" was published in 2021. Journal: Transl Neurosci.

Recently, research had found that the brain–spleen axis might contribute to the pathogenesis of depression [91]. In mice model of chronic social defeat stress (CSDS), natural killer group 2, member D (NKG2D) expression in the spleen, splenic volume, and weight in CSDS-susceptible mice were higher than that of control mice and CSDS-resilient mice. In addition, NKG2D expression in the spleen of patients with depression was higher than that in controls. Administration of (*R*)-ketamine could ameliorate the increased splenic weight and increased splenic NKG2D expression in CSDS-susceptible mice [91]. The brain–spleen axis provides a new research direction and target for ketamine in the treatment of depression.

As above, blocking NMDAR is a classic antidepressant mechanism of ketamine. Based on previous research, NMDARs are ionic receptors of glutamate, exiting on GABAergic inhibitory interneurons, extra-synaptic, intra-synaptic. Ketamine plays a role through four mechanisms of inhibiting NMDAR. First, ketamine selectively block NMDARs expressed on GABAergic inhibitory interneurons, leading to the release of glutamate receptors in synapses. Glutamate can activate AMDARs, thereby producing neuroprotective effect [81–84]. Second, ketamine inhibits extra-synaptic GluN2B-containing NMDARs, so as to prevent the tetanic activation of these receptors induced by peripheral glutamate. Third, ketamine blocks intra-synaptic NMDARs, which results in the inhibition of the eukaryotic elongation factor 2 kinase (eEF2K) activity, thus prevents eEF2 substrate phosphorylation and finally enhances BDNF translation. Fourth, ketamine inhibits NMDAR-dependent burst activity of neurons in lateral habenula nucleus [92]. There are two kinds of glial cells involved in this mechanism: microglia and astrocytes. The activation of microglia will produce quinolinic acid, which leads to excessive activation of NMDAR and excitotoxicity; astrocytes can take in extra synaptic glutamate, and if it is damaged, it will lead to excessive glutamate. We will mainly introduce the regulation of ketamine on these two kinds of cells.

### 5.1 Microglial

Studies have shown that chronic restraint stress induces depression-like behavior in mice, which is associated with microglial activation and upregulation of TLR4/p38 and P2X7 receptors in the hippocampus, and this neurobehavioral and biochemical abnormality is normalized by ketamine treatment [93]. Chronic unpredictable mild stress upregulates hippocampal IL-1β, IL-6, TNF-a, IDO, and KYN/tryptophan ratios, induces depression-like behavior, and subanesthesia doses of ketamine can reduce these inflammatory factors; therefore, its antidepressant effect is related to the downregulation of pro-inflammatory cytokines in rat hippocampus [94]. There are a large number of microglia in the hippocampus, and the increase in pro-inflammatory cytokines is related to the activation of microglia. Autopsy revealed an increase in the density of microglial cells producing quin in the anterior cingulate gyrus of depressed suicidal patients [95]. In LPS-induced depression-like mice model, a single dose of ketamine can improve depression-like behaviors and inhibit release of pro-inflammatory cytokines (IL-1α, IL-6, Eotaxin, G-CSF, MIP1b, and TNF-α) in the brain, attenuate morphological microglia reactivity and cytotoxic microglia polarization, reverse the overexpression of heme oxygenase 1 transcripts, and reduce the production of quin in microglia. In the conversion experiments of this study, plasma levels of metabolites in the KYN pathway of patients with MDD were abnormal. The KYNA/QUIN ratio before the first infusion is a predictive indicator of ketamine response, QUIN before each ketamine infusion is a biomarker of ketamine response, and the decrease in quin after ketamine infusion is a predictive indicator of decreased MADRS score. This study showed that microglia was a key target for ketamine therapy and quin was a biomarker of ketamine response in MDD [96]. In addition, ketamine may inhibit the overactivated microglia, reduce the release of pro-inflammatory cytokines, and enhance the release of anti-inflammatory cytokine IL-10 to improve depression [97–99]. A recent research which used HMC3 human microglial cell line showed that ketamine and its active metabolites, (2*R*,6*R*;2*S*,6*S*)-hydroxynorketamine (HNK), could regulate the type I interferon pathway mediated through STAT3 [100]. Specifically, ketamine and its active metabolite-regulated genes enriched in the “response to type I interferon”-signaling pathway. In the presence of ketamine and its active metabolites, STAT3 was translocated into the nucleus where it could act as a transcription factor. Furthermore, STAT3 mRNA nuclear expression was induced by exposure to them [100]. After STAT3 knockdown, ketamine or its active metabolites could not induce gene expression for type I interferon-signaling target genes [100]. It suggested that ketamine might play a role through type I interferon pathway in microglia, but it still needs to be verified *in vivo*.

The article "Immunoregulation and antidepressant effect of ketamine" was published in 2021. Journal: Transl Neurosci.

### 5.2 Astrocytes

Astrocytes are the most abundant cell type in the brain and are involved in homeostasis of the blood–brain barrier, axonal growth, and intracellular communication networks. Due to their altered expression and function in depression, astrocytes have recently received increasing attention. For example, Subjects with mood disorder had a decreased density of glial cells across all layers, and a reduction in astrocyte-specificmarker fibrillary acidic protein (GFAP) in white matter [101]. Pharmacological ablation of astrocytes in rat prefrontal cortex is sufficient to induce depression-like behavior [102]. Effective antidepressant treatment can inhibit the decrease in GFAP expression in patients with MDD. Astrocytes also secrete BDNF, a key molecule involved in the pathological process of MDD or the mechanism of antidepressants. Specific overexpression of BDNF in astrocytes produces anxiolytic-like activity [103]. Recently, there is a hypothesis that excessive NMDA receptors in astrocytes will lead to severe glutamate deficiency in MDD, and that ketamine-blocking excessive NMDAR in astrocytes may help to balance synaptic information processing [104]. Ketamine can significantly increase the expression of GFAP in the hippocampus. In addition, inhibition of astrocytes eliminated the antidepressant-like effects of ketamine in FST and TST. It is suggested that activated astrocytes play a vital role in the antidepressant activity of ketamine [105]. In order to determine whether the immunomodulatory effect of ketamine is related to its rapid antidepressant activity, cultured human astrocytes were incubated with ketamine, a mixture of cytokines or both, and ketamine dose dependently (100–500 μM) reduced production and gene expression of IL-6 and TNF-α within 24 h [106]. In addition, ketamine increases the density of cholesterol domains in the cytoplasmic membranes of astrocytes, which may be related to its antidepressant effect [107].

## 6 Conclusion

This study summarizes immune changes in MDD, the relationship between antidepressant therapy and immune regulation and describes how a novel antidepressant, ketamine plays an antidepressant role by regulating the immune mechanism. In addition to acting on its classic receptors and rapidly changing neuroplasticity, ketamine also improves depressive symptoms through immune regulation, including the regulation of peripheral cytokines and central glial cells. Immunomodulatory may be an important intermediate mechanism in antidepressant treatment of ketamine. Change of immune factors may become a biomarker to predict the responsiveness of ketamine to MDD, which provides a new direction for the treatment of TRD. However, these results are inconsistent and need further research. Moreover, there are still many clinical problems in the use of ketamine, such as possible tolerance, addiction, and psychotic side effects caused by overdose. Focusing on the immunomodulatory effect of ketamine may help to discover a new antidepressant mechanism of ketamine and develop more effective, safer, and more persistent antidepressants.

The article "Immunoregulation and antidepressant effect of ketamine" was published in 2021. Journal: Transl Neurosci.

## Abbreviations

AMPA: α-amino-3-hydroxy-5-methyl-4-isoxazolyl propionic acid
BDNF: brain-derived neurotrophic factor
CNS: central nervous system
CRP: C-reactive protein
CSDS: chronic social defeat stress
GFAP: fibrillary acidic protein
IDO: indoleamine-2,3-dioxygenase
IL: interleukin
INF: interferon
KYN: kynurenine
LBP: lipopolysaccharide-binding protein
LPS: lipopolysaccharide
MDD: major depressive disorder
NKG2D: natural killer group 2, member D
NMDAR: *N*-methyl-d-aspartate receptor
PBMC: peripheral blood mononuclear cell
P2X7R: purinergic ligand-gated ion channel 7 receptor
Quin: quinolinic acid
SSRIs: serotonin reuptake inhibitors
TH: T-helper
TLRs: toll-like receptors
TNF-α: tumor necrosis factor-α
TRD: treatment-resistant depression
